# Effect of Cold Fluid Compensatory Swallowing Combined with Balloon Dilation on the Treatment of Poststroke Cricopharyngeal Achalasia: A Pilot Randomized Controlled Trial

This article has been retracted.

**DOI:** 10.1155/2022/4171561

**Published:** 2022-10-08

**Authors:** Xiangwei Li, Linna Jin, Chengxiao Gu, Wangyuan Zhang, Xiao Zhou, Xiaoting You

**Affiliations:** ^1^Department of Rehabilitation, Hangzhou No. 128 Hospital, Hangzhou 310013, China; ^2^Department of Rehabilitation, Sir Runrun Shaw Hospital, School of Medicine, Zhejiang University, Hangzhou 310020, China; ^3^Department of Nursing, Hangzhou Anatorium of People's Liberation Army, Hangzhou 310013, China

## Abstract

**Objective:**

This study is aimed at comparing the treatment efficacy between catheter balloon dilation combined with cold fluid compensatory swallowing training and catheter balloon dilation alone on poststroke cricopharyngeal achalasia (CPA).

**Methods:**

We conducted a single-blind, randomized controlled trial (RCT). Poststroke patients with CPA were divided into two groups: the control group (treated with catheter balloon dilation) and the trial group (catheter balloon dilation combined with cold fluid compensatory swallowing). Videofluoroscopic swallowing study (VFSS) was performed, and functional oral intake scale (FOIS) was used to evaluate and compare the swallowing function of patients in the 2 groups before and after intervention. Posttreatment VAS pain scores and recovery time were also measured.

**Results:**

VFSS and FOIS scores in the two groups were improved after treatment (*P* < 0.05). In the trial group, VFSS scores in the pharyngeal phase and aspiration degree were significantly higher compared with the control group (*P* < 0.05) but not in the oral phase (*P* > 0.05). The difference in FOIS scores and patients' recovery time from intervention to eating mushy food between the trial and control groups was significant (*P* < 0.05), but not the VAS scores (*P* > 0.05).

**Conclusion:**

The catheter balloon dilation combined with cold fluid compensatory swallowing was superior to catheter balloon dilation alone in terms of relieving dysphagia and reducing aspiration in patients with CPA following stroke. Long-term efficacy should be followed up with more objective and quantitative indicators in future studies.

## 1. Introduction

The upper esophageal sphincter (UES), mainly comprised of cricopharyngeus muscle (CPM), is the gateway to the esophagus. CPM remains tightly closed to prevent air from entering the stomach and food reflux in the resting state. During swallowing, the CPM relaxes to allow the bolus to pass [1]. Cricopharyngeal achalasia (CPA) is characterized by incomplete relaxation of UES or lack of coordination of the UES opening with pharyngeal contractions [2]. It occurs when the CPM fails to relax during deglutition, and patients with CPA present symptoms such as swallowing dysfunction, dehydration, aspiration, choke and malnutrition, nasopharyngeal regurgitation, and respiratory illnesses, which seriously affect the life quality of patients [3, 4].

CPA is a typical dysphagia associated with stroke [5]. Lateral medullary lesion has been identified as an independent predictor for CPA [6]. Among patients suffering from brainstem stroke, the incidence of accompanying CPA is as high as 50% [7]. Effective protocols are needed for dysphagia management to avoid severe clinical complications and reduce morbidity and mortality of poststroke patients. Catheter balloon dilation is widely applied in clinic poststroke CPA treatment. The possible mechanism of the balloon dilatation for CPA treatment might be that the sensory input from the inflated balloon promotes the motor responses of the swallowing central pattern generator [8]. Balloon dilatation has the advantages of noninvasiveness, easy operation, and minor side effects [9, 10]. However, repeated catheterization and balloon pulling in balloon dilation may cause local mucosal edema and pain, resulting in poor tolerance and coordination [11]. Yuan and Zhang have reported the rehabilitation compliance of patients with dysphagia and cricopharyngeal dysfunction and proposed that balloon dilation therapy is more effective in patients with good adherence [12]. CPM can respond to oropharyngeal, esophageal, and neurohormonal triggers through complex control networks. Thus, even minor stimuli may change the behavior of CPM [6]. For example, transcranial magnetic stimulation on the motor cortex can produce motor evoked potential on the CPA and induce UES contraction [13]. Air and water stimulation induces lower esophageal sphincter relaxation accompanied with UES contractile reflex [14]. Ice packs have been used to reduce swelling and relieve pain. Studies have shown that ice stimulation can significantly shorten the swallowing reflex time, trigger swallowing movement, and enhance oropharyngeal muscular coordination [15]. It mainly increases sensory input to enhance the sensitivity of swallowing reflex by stimulating the soft palate and pharynx to sharpen the sensitivity of local nerve sensation and reconstructing the neurological network [16]. Therefore, it is indicated that ice stimulation may improve the motor and sensory activities of the cricopharyngeal muscle and promote the swallowing reflex. In addition, ice stimulation can reduce the incidence of aspiration, thereby improving patients' attention to feeding [17]. Studies [18, 19] have confirmed that ice water balloon dilatation can improve swallowing function and alleviate the adverse reactions caused by balloon dilation, which is of clinical significance.

However, there is insufficient evidence for the clinical efficacy of cold fluid compensatory swallowing. In this study, we aimed to explore the therapeutic efficacy of cold fluid compensatory swallowing combined with balloon dilation on swallowing function and quality of life of stroke patients with CPA. We hypothesized that combination with cold fluid compensatory swallowing could improve the swallowing function of patients compared with balloon dilation treatment alone. The findings of our study may provide novel strategy for the management of poststroke CPA.

## 2. Methods

### 2.1. Study Design and Subjects

This single-blind randomized trial recruited stroke patients treated at the Rehabilitation Department of in Hangzhou No. 128 Hospital, China, from December 2019 to February 2021. The inclusion criteria were as follows: (1) patients aged 18-80 years old, (2) stroke patients who met the national diagnostic criteria of cerebrovascular diseases through cranial CT or MRI [20], (3) videofluoroscopic swallowing study [21] (VFSS) confirmed achalasia of the cricopharyngeal muscle, and (4) Chinese version of Mini-Mental State Examination (MMSE) [22, 23] score ≥ 24. The exclusion criteria were as follows: (1) patients who underwent transnasal balloon dilatation; (2) unstable vital signs, failure of essential organs, and pregnant or lactating women; (3) previous abnormal structures of the oral cavity, pharynx, and esophagus; and (4) recent treatments or presence of previous or current conditions that might impact the results of the trial. This study was approved by the Clinical Research ethics committee of Hangzhou No. 128 hospital, China (no. 20200107-04). Informed consent was obtained from each patient. The study was registered in the Chinese Clinical Trial Registry (ChiCTR2200061770).

### 2.2. Intervention

According to the computer-generated randomization sequence, the included cases were randomly divided into the trial group (patients underwent catheter balloon dilation combined with cold fluid compensatory swallowing) and the control group (patients underwent catheter balloon dilation). One nurse generated the random allocation sequence, enrolled participants, and then assigned participants to interventions. The allocation sequence was concealed in numbered sealed opaque envelopes. The physicians and occupational therapists were blind to treatment allocation. Under the guidance of speech-language therapists, both groups completed routine swallowing function training [24], low-frequency electrical stimulation [24], and catheter balloon dilatation [8]. Regular swallowing function training included basic, direct, and compensatory training for 30 minutes per day, 5 days per week.

Trial group: patients held a urethral catheter (14Fr) in the mouth and actively swallowed it. When it is difficult to swallow the catheter, the rehabilitation nurse pushed the catheter appropriately, observed the response of patients, and then performed catheter balloon dilatation [8]. The process was repeated ten times, about 30 minutes each time, three times a week. After dilatation, patients continued to take ice water compensatory swallowing training [25]. They drank ice water with a long handle spoon at 4°C for 1 ml each time and swallowed with the head down and exerted force as instructed for about 15 minutes. The nurse affirmed the successful swallowing of patients.

Control group: after undergoing catheter balloon dilatation as the trial group, patients were given dexamethasone, chymotrypsin, and gentamycin nebulization to prevent mucosal edema and reduce mucus secretion.

### 2.3. Outcomes

All participants were initially evaluated for the severity of swallowing disorder with VFSS and FOIS before and after resuming oral feeding and after four weeks of treatment. One occupational therapist was trained to evaluate patients' VAS scores and average hospital stay after treatment.

### 2.4. Primary Endpoints

Videofluoroscopic swallowing study (VFSS) [21] evaluation: VFSS is the gold standard to diagnose and evaluate the swallowing function of patients with dysphagia. Philips Digital Gastrointestinal Machine was used for fluoroscopy acquisition. The video images were recorded with lateral projection and stored digitally at a speed of 30 frames per second. The swallow consistency order was thick-liquid, semisolid, solid, and thin-liquid. Based on angiography, the VFSS scores were assessed at three phases: oral phase (0-3 points), swallowing phase (0-3 points), and aspiration degree (0-4 points). For the oral phase, 0 point indicates nonswallow or swallow by gravity; 1 point indicates that no bolus formation, only flow of disperse food; 2 points indicate inadequate swallow with some remaining food in oral cavity; 3 points indicate a normal complete swallow at one time. For the swallowing phase, 0 point indicates no laryngeal elevation, closure of epiglottis and palatine arches, and inadequate swallow reflex; 1 point indicates large residue in pyriform sinus, 2 points indicate small amount of residue that can be repeatedly swallowed; 3 points indicates the adequate swallow. For the aspiration degree, 0 point indicates large aspiration without choke; 1 point indicates large aspiration with choke; 2 points indicate small amount of aspiration without choke; 3 points indicate small amount of aspiration with choke; 4 points indicate no aspiration. The VFSS scale covered 13 items, with a total score of 10 points. The higher the score was, the better the rehabilitation effect on swallowing function would be.

Functional oral intake scale (FOIS) [26]: according to the patients' oral feeding situation, the patients' swallowing function was evaluated by FOIS scoring into 7 grades from I to VII, corresponding to 1 to 7 points: I, nothing by mouth; II, tube feeding, with minimal attempts of food; and fluid; III, tube feeding, with consistent intake of food and fluid; IV, a total oral diet with a single consistency; V, a total oral diet with multiple consistencies that were specially prepared or compensated; VI, a total oral diet with multiple consistencies without special preparation, but with specific food limitation; and VII, a total oral diet with no restrictions. The FOIS score ≥ 3 was regarded as significant improvement.

### 2.5. Secondary Endpoints

Visual analogue scale (VAS) [27, 28]: VAS is a continuous scale self-completed by the respondent. It is usually comprised of a horizontal or vertical line at 10 cm long marked with verbal descriptors for extreme at both ends. Herein, we used a numeric version of VAS. The patients were asked with an introductory question and select a number ranging from 0 to 10 integers that best matched their pain intensity. It is an 11-point numeric scale representing different levels of pain, where 0 meant no pain (one extreme) and 10 meant extreme pain (the other extreme). The higher the score was, the more severe the pain patients suffered. We used VAS scores and visual evaluation to evaluate the adverse events, including mucosal edema, bleeding, and pain. Recovery time referred to the period from the first day of intervention to the day when the patient started to eat mushy food.

### 2.6. Sample Size

The sample size was calculated using the G∗Power 3.1.9 program based on a previous study [8]. The effect size of the repeated-measures analysis of variance was 0.3, with a power of 0.95 and a significance level of 0.05, using two groups and three rounds of measurements. The minimum sample size was 16 per group. A total of 36 participants were selected, with 18 participants in each group, accounting for a predicted dropout rate of 20%.

### 2.7. Statistical Analysis

Statistical analyses were performed using IBM SPSS 25.0. The measurement data were expressed as the mean ± standard deviation (SD). Independent *t*-test was used to compare numerical parameters between two groups. Independent sample *t*-test was used for intergroup comparison, and paired sample *t*-test was used for intragroup comparison. Statistical significance was set at *P* < 0.05.

## 3. Results

In this study, we evaluated the effect of cold fluid compensatory swallowing combined with balloon dilation compared with catheter balloon dilation alone on the treatment of poststroke CPA patients using a randomized controlled trial. We found that the trial group presented higher efficacy to relieve dysphagia and aspiration in the pharyngeal phase and aspiration degree compared with the control group, improving the swallowing function and promoting the recovery of patients with CPA post stroke.

### 3.1. Participants

Following the inclusion criteria and exclusion criteria, 36 patients were included. The study flowchart is presented in Figure 1.

The clinical characteristics of patients enrolled in this study were shown in Table 1. There was no significant difference in general data, such as gender, age, stroke duration, stroke type, lesion location, and degree of dysphagia and pain, between the two groups. One patient in the trial group dropped out for personal reasons.

### 3.2. VFSS and FOIS Scores

VFSS and FOIS scores in the two groups were both elevated after treatment (both *P* < 0.05) (Tables 2 and 3). Compared with the control group, VFSS scores were significantly increased in the pharyngeal phase and aspiration phase (both *P* < 0.05), but not in the oral phase (*P* > 0.05) in the trial group. FOIS scores in the trial group were higher than those in the control group and showed significant increase in the trail group after the treatment (*P* < 0.05).

### 3.3. Recovery Outcome

After intervention, 16 patients in both groups recovered and began to eat food, and 3 patients still could not eat even the mushy food. The differences in patients' recovery time from eating meals between the trial and control groups were significant, and patients in the trial group had shorter recovery time compared with the control group (both *P* < 0.05), whereas VAS score showed no significant difference between the two groups (*P* > 0.05) (Table 3).

## 4. Discussion

This study indicated significant differences in VFSS scores of swallowing period, degree of aspiration, and FOIS scores between catheter balloon dilation combined with cold fluid compensatory swallowing training and catheter balloon dilation alone for the treatment of poststroke cricopharyngeal achalasia patients (*P* < 0.05). The combination treatment can improve swallowing function and reduce pulmonary infection, which was consistent with the research by Zhuang et al. [18]. Compared with the previous study, we used both VFSS and FOIS scoring systems to evaluate the swallowing function of patients. The effects were compared before and after treatments as well as between the control and trial groups to achieve a valid conclusion. Catheter balloon dilatation is widely used in the treatment of dysphagia caused by CPA [10]. During swallowing, the expanded balloon stretches the CPM to promote its opening, stimulates the CPM with a certain sense of tactile and pressure, and induces reflex swallowing through the superior laryngeal nerve to regulate the excitability of the brainstem swallowing center [8]. There are various sensory receptors in the mouth and pharynx. Sensory input plays a critical role in the initiation and regulation of swallowing [29]. After balloon dilatation, the patients in the trial group swallowed cold liquids with their heads down to consolidate the therapeutic effect of balloon dilatation on the swallowing muscle groups. The rehabilitation specialist nurse observed the patient's response, provided timely guidance, and gave positive affirmation and feedback. Studies [30, 31] have revealed that repeated ice stimulation increases the excitability of the cortical swallowing motor pathway, which is beneficial to rebuild the neural function network between the cortex and the medulla and restores the cortical regulation of the brainstem swallowing center. Drinking ice water can shorten the pharyngeal reaction time, prolong the laryngeal elevation time, and accelerate the laryngeal closure speed [30, 31]. Pharyngeal cold stimulation can effectively improve the sensitivity of the soft palate and pharynx, make swallowing easier, attract patients' attention on feeding and swallowing, and reduce aspiration. Li et al. [32] have found that patients who receive ice stimulation training experience less adverse events (e.g., aspiration, choking, and aspiration pneumonia) compared with the control group, and the difference was statistically significant. Compared with the previous studies, we combined the ice stimulation and catheter balloon dilation for the treatment of poststroke patients with CPA. We found ice stimulation improved the treatment efficacy compared with the catheter balloon dilation alone, which relieved dysphagia and aspiration in the pharyngeal phase and aspiration degree and promoted the recovery of swallow function of patients.

Our study also showed significant differences in patients' recovery time from intervention to eating meals between the trial and control groups (*P* < 0.05), but VAS scores showed no difference between the two groups (*P* > 0.05). The reason might be that patients in the control group were given dexamethasone, chymotrypsin, and gentamycin nebulization after dilatation, preventing mucosal edema and reducing mucus secretion. The pain of patients in both groups was controlled. Successful experience can improve patients' self-efficacy [33], which makes patients more actively coordinated. Our study enables patients to continuously practice near-physiological swallowing, enhancing patients' self-confidence by successfully drinking cold liquids and making them more cooperated with active swallowing catheter insertion before balloon dilation. Active swallowing catheter insertion can also help repeatedly train the muscles, improving their strength and coordination of swallowing muscle groups [34]. Swallowing catheter placement consolidates and improves the role of catheter balloon dilatation in treating CPA and promotes the recovery of patients' swallowing function. Yang et al. [16] compare the efficacy of ice water balloon dilatation with regular temperature balloon dilatation. They find that the differences in average treatment times, average hospital stay, and average treatment cost between the two groups are noticeable. Ice water balloon dilatation is more effective (*P* < 0.05), which is in line with the findings by Sun and Wang [35]. One study has reported [18] that ice water alleviated and controlled pharyngeal pain, congestion, and edema caused by balloon expansion. We found that in the trial group, intervention relieved patients' discomfort and shorten the dysphagia treatment time. Compared with the previous studies, we conducted a randomized controlled trial to explore the effect of cold fluid compensatory swallowing combined with balloon dilation on the treatment of poststroke CPA patients. We used not only FOIS scores but also the gold standards methods such as VFSS to evaluate the swallow function recovery of patients. Ice stimulation has been demonstrated to promote the relaxation of CPA, which may effectively improve the treatment effect of catheter balloon dilation and accelerate the recovery of patients.

This study also showed no significant difference in VFSS scores between the two groups in the oral phase (*P* > 0.05) that might be related to the fact that the oral problems of the included patients were not prominent, and the retardation of the cricopharyngeal muscle mainly caused dysphagia. Moreover, this study still had some limitations. First, this was a single-blind trial with small sample size, and there was a lack of long-term efficacy follow-up. Second, our study used the VFSS and FOIS scores to clinically evaluate the swallowing function, which might be affected by subjective factors. We plan to evaluate swallowing process with more objective and quantitative indicators in future studies. Third, the adverse events, including mucosal edema, bleeding, and pain, were assessed through visual evaluation and VAS scores.

In conclusion, catheter balloon dilatation combined with ice water compensatory swallowing training may effectively improve the swallowing function and reduce aspiration of patients with CPA after stroke, relieve patients' throat pain, and shorten the treatment time. The findings of our study may provide a novel strategy for the management of poststroke CPA. In the future, we can further carry out the multicenter, large sample, long-term double-blind, randomized controlled research, to explore the relevant underlying mechanism, improve the training and treatment scheme, and provide a scientific and standardized reference basis for clinical treatment of poststroke CPA. Moreover, the evaluation systems should be optimized, and long-term treatment efficacy and recovery will be further explored in the future research.

## Figures and Tables

**Figure 1:** The study flowchart.

**Table 1:** Clinical characteristics of patients.

	Control group (*n* = 18)	Trial group (*n* = 18)	*P* value
Gender (M/F)	12/6	10/8	
Age (years)	62.22 ± 10.75	64.94 ± 10.22	0.442
Diagnosis			
Infarction	12	11	
Hemorrhage	6	7	
Time from onset (days)	45.83 ± 14.24	44.89 ± 15.73	0.851
Location			
Brain stem	10	12	
Combine	8	6	
Achalasia			
Complete	9	7	
Incomplete	9	11	
History			
Hypertension	17	16	
Diabetes	11	15	
Coronary heart disease	3	1	

**Table 2:** Comparison of VFSS scores between two groups.

VFSS	Group	Pretherapy	Posttherapy	95% confidence interval of the difference		*P* value
The oral phase	Control group	2.44 ± 0.51	2.61 ± 0.50	Low lever	High lever	
	Trial group	2.18 ± 0.53	2.35 ± 0.61	-0.124	0.640	0.178

Pharyngeal phase	Control group	1.50 ± 0.51	2.06 ± 0.54^a^	-0.877	-0.071	0.023
	Trial group	1.41 ± 0.50	2.53 ± 0.62^ab^			

Aspiration phase	Control group	2.56 ± 0.51	3.33 ± 0.48^a^	-0.701	-0.044	0.027
	Trial group	2.82 ± 0.53	3.71 ± 0.47^ab^			

Total	Control group	6.44 ± 1.04	8.39 ± 0.78^a^	-0.745	0.700	0.949
	Trial group	6.82 ± 1.01	8.41 ± 1.28^a^			

**Table 3:** Comparisons of FOIS and VAS scores and recovery time between two groups.

	Group	Pretherapy	Posttherapy	95% confidence interval of the difference		*P* value
FOIS	Control group	1.72 ± 0.67	4.39 ± 0.98^a^	Low lever	High lever	
	Trial group	1.82 ± 0.73	5.18 ± 1.07^ab^	-1.496	-0.079	0.030

VAS	Control group		0.61 ± 0.70	-0.255	0.654	0.379
	Trial group		0.41 ± 0.62			

Recovery time (d)	Control group		26.13 ± 2.53	0.063	4.187	0.043
	Trial group		24.00 ± 3.14^b^			

Note: intragroup comparison before and after treatment, ^a^*P* < 0.05; compared with the control group after treatment, ^b^*P* < 0.05. d: days.

## Data Availability

The datasets used and analyzed in the current research would be available from the corresponding author upon request.
